# Tanshinone IIa Induces Autophagy and Apoptosis via PI3K/Akt/mTOR Axis in Acute Promyelocytic Leukemia NB4 Cells

**DOI:** 10.1155/2021/3372403

**Published:** 2021-10-15

**Authors:** Yiming Pan, Lingyan Chen, Ruibai Li, Yu Liu, Mengdie Nan, Li Hou

**Affiliations:** ^1^Department of Hematology and Oncology, Dongzhimen Hospital, Beijing University of Chinese Medicine, Beijing 100700, China; ^2^Zhejiang Provincial Key Laboratory of Medical Genetics, School, Laboratory Medicine and Life Sciences, Wenzhou Medical University, Wenzhou 325035, Zhejiang, China

## Abstract

Tanshinone IIa (TanIIa), an ingredient of Radix Salviae Miltiorrhizae, has an anticancer effect on various solid tumors with high efficiency and low toxicity. Nonetheless, the underlying role of TanIIa in acute promyelocytic leukemia (APL) remains unclear. Here, we revealed that TanIIa drastically inhibited NB4 cell viability with an IC50 value of 31.25 *μ*mol/L. Using flow cytometry apoptosis assay, we identified that TanIIa dose-dependently exacerbated NB4 cell apoptosis. Mechanistically, TanIIa upregulated apoptotic factor levels, namely, cleaved-caspase 9, cleaved-caspase 3, and cleaved-PARP-1. Moreover, we noticed that TanIIa dose-dependently suppressed the PI3K/Akt/mTOR axis. This axis not only functions as an essential antiapoptotic modulator but also serves as a suppressant regulator of autophagy. Correspondingly, we detected the levels of autophagic marker, namely, LC3B, which were increased after the TanIIa treatment. Furthermore, the autophagy inhibitor Baf-A1 could effectively reverse the TanIIa-induced apoptosis, manifesting that TanIIa eliminated NB4 cells in an autophagy-dependent manner. In conclusion, tanshinone IIa exerts anti-APL effects through triggering autophagy and apoptosis in NB4 cells.

## 1. Introduction

Characterized by severe coagulation abnormalities, acute promyelocytic leukemia (APL) was considered the most threatening leukemia subtype for decades before the prevalent application of arsenic trioxide (ATO) and all-trans retinoic acid (ATRA) [1]. Fortunately, ATO plus ATRA can surely elevate APL curative rate [1]. Nonetheless, roughly 10% of APL patients suffer a relapse owing to the insensitivity to ATO plus ATRA regimens [2–4]. What is more serious is that the 3-year survival rate for people with relapsed APL is only 50–70% [5, 6]. Therefore, there is still a crying need to find novel and effective drugs for APL.

Radix Salviae Miltiorrhizae, the dried rhizome and root of the plant *Salvia miltiorrhiza* Bge, is a traditional herb that is frequently utilized in the treatment of cancers, cardiovascular diseases, and neurodegenerative diseases [7, 8]. Tanshinone IIa (TanIIa; 1,6,6-trimethyl-8,9-dihydro-7H-naphtho[1,2-g][1]benzofuran-10,11-dione; Figure 1(a)), the main composition extracted from the Radix Salviae Miltiorrhizae, has demonstrated efficient anticancer effects in solid tumors, such as lung cancer, gastric cancer, pancreatic cancer, ovarian cancer, cervical cancer, and colorectal cancer [9]. Previous studies implied that TanIIa exerts anticancer effects through various approaches, including promoting apoptosis, inducing autophagy, and mediating cell cycle arrest [9].

The PI3K/Akt/mTOR axis functions as a primary antiapoptotic modulator that promotes cellular survival and reduces cellular death in response to external stress, as well as serves as a suppressant regulator of autophagy [10]. Anomalous activation of PI3K/Akt/mTOR axis contributes to the unconstrained proliferation of cancer cells and is the most commonly occurring pathway anomalies involved in the maintenance and progression of numerous cancers [11, 12]. Therefore, inhibiting PI3K/Akt/mTOR axis has been disclosed as a promising therapeutical goal for cancers. When it comes to acute myelocytic leukemia (AML), more than half of the patients are identified with the same disorder of PI3K/Akt/mTOR axis, which contributes to the decreased long-term survival [13]. Unsurprisingly, blocking PI3K/Akt/mTOR axis compels AML cells towards apoptosis resulting in enhanced therapeutic outcomes of chemotherapy [14–17].

As the primary cellular mechanism for recycling proteins, autophagy occurs in response to adverse stimuli to relieve metabolic stress and stabilize the internal environment [18]. However, excessive autophagy under certain circumstances can trigger autophagic death, namely, type II programmed cell death for the threshold of the protective effect is exceeded [19]. Autophagic death can occur simultaneously with apoptosis, which in turn accelerates the speed of cancer cell death [20–22]. Therefore, stimulation of autophagy can be used as a potential approach to treat cancers [23]. Interestingly, the reaction of APL cells to ATO plus ATRA treatment is autophagy-dependent, while blocking autophagy damages the therapeutic effect [24].

In conclusion, we believe that TanIIa has potential in treating APL, but its effect on APL has not been well studied. Here, we studied the anti-APL effects of TanIIa so that a therapeutic alternative will be developed.

## 2. Reagents and Methods

### 2.1. Reagents

Tanshinone IIa (purity ≥99%, HY-N0135) and bafilomycin A1 (HY-100558) were purchased from MedChemExpress, Inc. IMDM medium (12440061) and fetal bovine serum (10099141) were purchased from Gibco, Inc. Primary antibodies: anti-caspase-9 (32503), anti-caspase-3 (32351), anti-PARP-1 (191217), anti-mTOR (2732), anti-phosphorylation-mTOR (109268), anti-phosphorylation-ULK-1 (203207), anti-LC3B (192890), and anti-*β*-actin (8226) were purchased from Abcam, Inc.; anti-PI3K (13666), anti-phosphorylation-PI3K (17366), anti-Akt (4685), and anti-phosphorylation-Akt (4060) were purchased from Cell Signaling Technology, Inc. Giemsa Stain Solution (G1015) was purchased from Solarbio Life Sciences, Inc. CCK-8 kit (CK04) was purchased from Dojindo Molecular Technologies, Inc. Apoptosis kit with Annexin V/PI staining (556547) was purchased from BD Biosciences, Inc.

### 2.2. Cell Culture

Human APL cell line NB4 was generously gifted by Professor Yang Shen of Ruijin Hospital, Shanghai Jiao Tong University. NB4 cells were maintained in the IMDM medium supplemented with 10% fetal bovine serum and cultured in a humidified incubator at 37°C under a 5% CO_2_ atmosphere.

### 2.3. Cell Viability and Proliferation Assay

The CCK-8 kit was utilized to quantify the changes in cell viability and proliferation after TanIIa treatment. Experiments were all carried out using 96-well plates. NB4 cell suspension density was adjusted to 4 × 10^4^ cells/mL, and then we added 0.1 mL suspension to every well. After the seeding, NB4 cells were treated with 0, 1, 2, 4, 8, 16, 32, 64, 128, and 256 *µ*mol/L TanIIa for 24 h. 10 *μ*L CCK-8 was added to each well and incubated for 1–4 h under light-proof conditions. The optical density at 450 nm of wells was quantified by the Varioskan™ LUX multiplate reader. For the cell proliferation assay, 2 × 10^3^ NB4 cells were transferred into wells and treated with 0, 16, 32, and 64 *µ*mol/L TanIIa for 0–72 h. After the treatment, the relative cell number was obtained by CCK-8 analysis.

### 2.4. Giemsa Staining

Morphological alteration of NB4 cells was studied via Giemsa staining. Treated NB4 cells were washed with PBS and resuspended with FBS to prepare cellular slides. These slides were fixed with methanol for 5 min and then treated with Giemsa staining solution for 10–15 min. Stained slides were rinsed in running water and dried naturally. Stained slides were placed under the light microscope and observed at a magnification of 400×.

### 2.5. Annexin V/PI Staining Assay

The percentage of apoptotic cells is obtained via flow cytometry analysis after staining the cells with Annexin V/PI. The treated NB4 cells were collected and washed with precooled PBS. The cells were resuspended by adding 0.1 mL of 1× binding buffer with gentle blowing. 5 *μ*L PI and Annexin V were added to each sample and incubated for 15 min at room temperature under light-proof conditions, and then we added 0.4 mL of 1× binding buffer to decrease the density to improve assay accuracy. Cells were assayed for apoptosis using flow cytometry (BD Accuri™ C6 Plus).

### 2.6. Western Blotting

Cell precipitate was collected after the treatment and washed at least 2 times with precooled PBS. The cell precipitate was digested with RIPA lysate and centrifuged to obtain a protein-rich supernatant. The protein supernatant was adjusted to a concentration of 1 *μ*g/mL using 2× loading buffer. During sample loading, we made sure that each sample contained the same amount of total protein. Sample proteins were separated in SDS-PAGE at 120 V and transferred from the SDS-PAGE onto the nitrocellulose membrane at 100 V. Nitrocellulose membranes are blocked in 5% skimmed milk for 2 h. Samples were incubated with primary antibody overnight at 4°C and secondary antibody for 1 h at room temperature. The proteins were visualized with ECL. Protein expression levels were quantitated via ImageJ software.

### 2.7. Statistical Analysis

All experiments in this study were performed at least three times. Comparisons between the two groups were analyzed by using Student's *t*-test, and the graphs were created by GraphPad 7.0 software. *P* < 0.05 was considered a statistically significant difference. All data were expressed as the mean ± SD.

## 3. Results

### 3.1. TanIIa Inhibited NB4 Cell Viability and Proliferation

To evaluate the anti-APL activity of TanIIa on NB4 cells, we performed cellular viability and proliferation assays via the CCK-8 assay. We treated NB4 cells with different doses of TanIIa for 24 h. With the increasing of TanIIa doses from 1 *μ*mol/L to 256 *μ*mol/L, it gradually inhibited NB4. Of note, the IC50 was 31.25 *μ*mol/L (Figure 1(b)). We analyzed the proliferation rate of NB4 cells treated with different doses (0, 16, 32, and 64 *μ*mol/L) and different times (0, 24, 48, and 72 h) of TanIIa using the CCK-8 assay (Figure 1(c)). The results manifested that TanIIa markedly suppressed NB4 proliferation via dose-dependent and time-dependent manners (Figure 1(c)).

### 3.2. TanIIa Prompted Apoptosis in NB4 Cells

Through Giemsa staining, we found that 16 *µ*mol/L TanIIa increased the proportion of apoptotic cells in comparison to the 0 *μ*mol/L groups. Furthermore, NB4 cells treated with 32 and 64 *µ*mol/L TanIIa exhibited the morphology of late apoptosis which manifested itself in cytoplasmic condensation, nuclear condensation, or nuclear fragmentation (Figure 2(a)). Apoptosis analysis showed that the percentage of apoptotic cells in the 0 *µ*mol/L group was 3.60%, while the percentage in 16, 32, and 64 *μ*mol/L TanIIa-treated groups increased to 14.58%, 23.4%, and 39.3%, respectively (Figure 2(b)). Observing the changes in apoptosis-related factors through western blotting, we noticed that TanIIa enhanced the cleavage of caspase-9, caspase-3, and PARP-1 in NB4 cells (Figure 2(c)). Therefore, these results indicated that the antiproliferative effects of TanIIa could be accelerated by its apoptosis-inducing propensity in NB4 cells.

### 3.3. TanIIa-Induced Autophagy via PI3K/Akt/mTOR Axis in NB4 Cells

In addition to acting as an antiapoptotic regulator, the PI3K/Akt/mTOR axis also has a role in inhibiting cellular autophagy which can be induced by inhibiting the signal transduction of this axis. The impact of TanIIa exposure on the PI3K/Akt/mTOR axis and autophagy in NB4 cells was analyzed through western blotting. Treated with variant doses, namely, 0–64 *µ*mol/L of TanIIa, the levels of p-ULK-1 and LC3B increased while the PI3K, Akt, and mTOR protein levels and their phosphorylation levels significantly decreased (Figure 3). These results indicated that TanIIa inhibited the PI3K/Akt/mTOR axis and induced autophagy in NB4 cells.

### 3.4. Blocking of Autophagy Reduced Apoptosis Induced by TanIIa

Autophagy is a biological behavior in which cells undergo self-cannibalization, digestion to recycle abnormal and damaged biomolecules in response to various stimuli, maintaining the stability of the internal environment to sustain their survival. Although autophagy fights against various adverse factors, it also causes excessive self-digestion and then triggers autophagic death, a kind of programmed cell death, which is usually accompanied by apoptosis. Therefore, inhibiting or activating autophagy is considered as a promising approach for both cancer prevention and treatment. To investigate the effect of autophagy on TanIIa-induced cytotoxicity in NB4 cells, we used a classical autophagy inhibitor bafilomycin A1 (Baf-A1) to block the TanIIa-induced autophagy. Then, we detected the apoptosis rate of NB4 cells after treating with Baf-A1 by using Annexin V/PI assay and western blotting. As expected, we found that Baf-A1 did not induce significant cytotoxicity on NB4 cells (Figure 4(a)). Meanwhile, TanIIa combined with Baf-A1 attenuated TanIIa-triggered apoptosis in NB4 cells (Figure 4(b)). Therefore, our results demonstrated that TanIIa-induced autophagy played an apoptosis-promoting role on NB4 cells.

## 4. Discussion

APL is a common subtype of AML with t(15;17) chromosomal translocation triggering a PML-RAR*α* rearrangement as the characteristic genetic event and is considered the most aggressive and fatal subtype of AML [1]. PML-RARA fusion protein causes differentiation arrest of hematopoietic progenitor cells at the promyelocytic stage and confers resistance to apoptosis, ultimately developing into APL [1]. ATO plus ATRA has greatly improved the prognosis of APL, but about 10% of patients will relapse owing to resistance to ATO plus ATRA [2–4]. Beyond well-controlled clinical trials, the prognosis of APL is not as good as we expect [25]. Therefore, curing all APL patients remains a challenge currently for us and it is still significant to explore new treatment strategies or find alternative drugs.

As a natural substance with hypotoxicity, TanIIa is popularly used in China as adjuvant therapy for cardiovascular diseases [7, 8]. Numbers of research focused on TanIIa have shown its anticancer effect in various solid tumors via inhibiting cell growth and promoting cell apoptosis [9]. A male patient with relapsed APL resistant to ATO plus ATRA achieved morphologically complete remission after treatment with TanIIa at West China Hospital, and no significant toxic side effects were observed during TanIIa treatment [26]. This case report reveals the potential of TanIIa in the induction therapy for APL. Considering that the effectiveness of TanIIa against APL is not well studied, we observed the antiproliferative and proapoptotic activity of TanIIa on NB4 and further explored the mechanism.

By using CCK-8 assay and flow cytometry apoptosis analysis, we revealed that TanIIa exhibited the anti-APL effect via inhibiting proliferation as well as promoting apoptosis. Apoptosis is identified as the most primary form of cell death and is mediated by two main apoptotic pathways, namely, intrinsic and extrinsic apoptosis pathways [27]. The intrinsic apoptosis pathway is launched by augmenting the permeability of mitochondria and extricating cytochrome C into the cytoplasm, which further activates downstream caspase-9 and caspase-3 to execute apoptotic cell death [28]. PARP-1 is essential for DNA repair and plays a crucial part in maintaining cell survival; therefore, the cleavage of PARP-1 caused by cleaved-caspase-3 hampers DNA repair, compels cells towards death, and consequently serves as an indicator of apoptosis [29]. Western blot analysis exhibited that the cleavage of caspase-3, caspase-9, and PARP-1 was significantly upregulated after TanIIa treatment. These phenomena suggested that TanIIa induced NB4 cell apoptosis through the intrinsic apoptosis pathway.

The PI3K/Akt/mTOR axis, the most commonly hyperactivated pathway of human cancers, plays a pivotal role in promoting cell growth, proliferation, and survival and acting as a negative regulator of autophagy [30]. Serving as an antiapoptotic regulator, the hyperactivation of PI3K/Akt/mTOR axis prevents the initiation of intrinsic pathway mediated apoptosis by phosphorylating downstream Bax and Bad, provoking resistance to apoptotic signals of cancer cells [31]. Correspondingly, the blockage of PI3K/Akt/mTOR axis promotes the expression of Bax, caspase-9, and caspase-3, which initiates intrinsic signaling pathway mediated apoptosis [32]. Likewise, the suppression of PI3K/Akt/mTOR axis exerts antileukemia effects and enhances chemosensitivity through inducing autophagic cell death and apoptosis in vitro [33, 34]. In our study, treatment with TanIIa decreased the activation of PI3K/Akt/mTOR axis dose-dependently, suggesting that TanIIa-triggered intrinsic apoptosis is associated with the suppression of PI3K/Akt/mTOR axis.

In addition, we noticed that the suppression of PI3K/Akt/mTOR axis was accompanied by an increase in LC3B which is a marker of autophagy. To confirm that the autophagy that occurred in NB4 cells after TanIIa treatment was a manifestation of autophagic death caused by blockage of PI3K/Akt/mTOR rather than a self-protective stress response, we performed further experiments using Baf-A1. Baf-A1, a small-molecule inhibitor of vacuolar H^+^-ATPase, obstacles autophagosome-lysosome fusion and acidification of lysosomes in treated cells [35]. We found that coadministration of Baf-A1 markedly reduced the anti-APL effect of TanIIa, suggesting that autophagy triggered by TanIIa is a manifestation of autophagic death and acts as a component of its anti-APL effect.

Autophagy is an important approach for intracellular degradation of biomolecules by sequestering abnormal or damaged proteins and organelles in autophagosomes and fusing with lysosomes, leading to the degradation of the sequestered biomolecules into the recyclable small-molecule organic matter [36]. In most cases, autophagy plays a role in stabilizing the internal environment to promote cancer cell survival and only in some conditions exerts a therapeutic effect in the form of programmed death II [36]. However, emerging studies suggest that activation of autophagy is a potent therapeutic target of AML. Autophagy plays an important part in the maturation of myeloid progenitor cells, and inhibiting autophagy causes defective differentiation [37]. As a negative modulator of autophagy, the hyperactivation of PI3K/Akt/mTOR axis leads to the inactivation of autophagy in AML cells and is vital for maintaining the oncogenic potential of leukemia stem cells [38, 39]. Blocking autophagy reduces the efficacy of ATO plus ATRA on NB4 cells [38]. Suppressing the PI3K/Akt/mTOR axis via Akt inhibitors promotes programmed death in APL [40, 41].

Recent reports suggested that the regulatory effect of TanIIa on the PI3K/Akt/mTOR axis is not confined to APL. Zhang et al. showed that TanIIa caused autophagy and apoptosis in acute monocytic leukemia cells by downregulating the PI3K/Akt axis [42]. Liu et al. revealed that TanIIa inhibited glycolysis and induced apoptosis in cervical cancer cells by blocking the Akt/mTOR axis [43]. Wang et al. indicated that TanIIa reverses gefitinib resistance in lung cancer cells by downregulating VEGFR/Akt axis [44]. Wang et al. reported that TanIIa in combination with astragaloside IV exerted a stabilizing effect on atherosclerotic plaques by modulating the Akt signal [45]. Tanshinone I is another ingredient extracted from Radix Salviae Miltiorrhizae. Zhou et al. found that tanshinone I dose-dependently suppressed the PI3K/Akt/mTOR axis and triggered autophagy and apoptosis in ovarian cancer cell lines [46]. Considering that the PI3K/Akt/mTOR axis is a therapeutic target for many diseases, especially cancers, we believe it is meaningful to delve into research in TanIIa and other active substances of Radix Salviae Miltiorrhizae.

In conclusion, tanshinone IIa considerably compelled NB4 cells towards apoptosis via suppressing the PI3K/Akt/mTOR axis and activating the intrinsic apoptotic pathway. Tanshinone IIa also induced autophagy in NB4 cells, which enhanced the anti-APL effect. These results suggested that tanshinone IIa may be a complementary and alternative option for APL treatment.

## Figures and Tables

**Figure 1:** TanIIa inhibited NB4 viability and proliferation. (a) The chemical structure of TanIIa. (b) Cell viability assay: relative cell viability analyzed by CCK-8 in NB4 cells treated with different TanIIa doses, namely, 0, 1, 2, 4, 8, 16, 32, 64, 128, and 256 µmol/L for 24 h. Data were expressed as the mean ± SD of three independent experiments. (c) Cell proliferation assay: the relative cell number analyzed by CCK-8 in NB4 cells treated with TanIIa for 0–72 h. Data were expressed as the mean ± SD of three independent experiments.

**Figure 2:** TanIIa-induced NB4 apoptosis. (a) Giemsa staining of NB4 cells treated with TanIIa for 24 h. (b) Annexin V/PI staining of NB4 cells treated with TanIIa for 24 h. (c) The western blotting of apoptotic proteins in NB4 cells treated with TanIIa for 24 h. (d) The relative quantification of apoptotic proteins in NB4 cells treated with TanIIa for 24 h. Data were expressed as the mean ± SD of three independent experiments; ^*∗*^*P* < 0.05,  ^*∗∗*^*P* < 0.01,  and ^*∗∗∗*^*P* < 0.001, compared with the 0 *μ*mol/L groups.

**Figure 3:** TanIIa suppressed the PI3K/Akt/mTOR axis and activated autophagy in NB4 cells. (a) The western blotting of autophagic proteins in NB4 cells treated with TanIIa for 24 h. (b) The relative quantification of autophagic proteins in NB4 cells treated with TanIIa. Data were expressed as the mean ± SD of three independent experiments,  ^*∗*^*P* < 0.05, ^*∗∗*^*P* < 0.01,  and  ^*∗∗∗*^*P* < 0.001, compared with the 0 *μ*mol/L groups.

**Figure 4:** Blocking autophagy reduced the anti-APL effect of TanIIa. (a) The Annexin V/PI staining of NB4 cells treated with TanIIa or Baf-A1 or both for 24 h. (b) The western blotting of autophagic proteins in NB4 cells treated with TanIIa or Baf-A1 or both for 24 h. (c) The relative quantification of autophagic proteins in NB4 cells treated with TanIIa or Baf-A1 or both for 24 h. Data were expressed as the mean ± SD of three independent experiments,  ^*∗∗*^*P* < 0.01,  and  ^*∗∗∗*^*P* < 0.001, compared with the 0 *μ*mol/L groups.

## Data Availability

The data supporting the findings of the study are available from the corresponding author upon request.

## Abbreviations

Akt: Protein kinase B
AML: Acute myeloid leukemia
APL: Acute promyelocytic leukemia
ATO: Arsenic trioxide
ATRA: All-trans retinoic acid
Bad: Bcl-2-associated death promoter
Bax: Bcl-2-associated *X* protein
Caspase: Cysteinyl aspartate specific proteinase
IC50: Half maximal inhibitory concentration
LC3B: Microtubule-associated protein 1 light chain 3B type
mTOR: Mammalian target of rapamycin
p-Akt: Phosphorylated Akt
PARP-1: Poly(ADP-ribose) polymerase-1
PI3K: Phosphatidylinositol 3-kinases
PML: Promyelocytic leukemia protein
p-mTOR: Phosphorylated mTOR
p-PI3K: Phosphorylated PI3K
RAR*α*: Retinoic acid receptor *α*.
